The article "Recent Demographic History and Present Fine-Scale Structure in the Northwest Atlantic Leatherback (Dermochelys coriacea) Turtle Population" was published in 2013. Journal: PLoS One.

# Recent Demographic History and Present Fine-Scale Structure in the Northwest Atlantic Leatherback (*Dermochelys coriacea*) Turtle Population

**DOI:** 10.1371/journal.pone.0058061

**Published:** 2013-03-13

**Authors:** Érica Molfetti, Sibelle Torres Vilaça, Jean-Yves Georges, Virginie Plot, Eric Delcroix, Rozen Le Scao, Anne Lavergne, Sébastien Barrioz, Fabrício Rodrigues dos Santos, Benoît de Thoisy

**Affiliations:** 1 Departamento de Biologia Geral, ICB, Universidade Federal de Minas Gerais, 31270-010, Belo Horizonte, Minas Gerais, Brazil; 2 Dipartimento di Biologia ed Evoluzione, Sezione di Biologia Evolutiva, Università di Ferrara, Ferrara, Italy; 3 Université de Strasbourg, IPHC (Institut Pluridisciplinaire Hubert Curien), 67087, Strasbourg, France; 4 CNRS,UMR 7178, 67087, Strasbourg, France; 5 Office National de la Chasse et de la Faune Sauvage Guadeloupe, 97129, Lamentin, Guadeloupe, French West Indies; 6 Office National de la Chasse et de la Faune Sauvage, Martinique, 97200, Martinique, French West Indies; 7 Institut Pasteur de la Guyane, 97300, Cayenne, French Guiana; 8 Kwata NGO, 97300 Cayenne, French Guiana; Tuscia University, Italy

## Abstract

The leatherback turtle *Dermochelys coriacea* is the most widely distributed sea turtle species in the world. It exhibits complex life traits: female homing and migration, migrations of juveniles and males that remain poorly known, and a strong climatic influence on resources, breeding success and sex-ratio. It is consequently challenging to understand population dynamics. Leatherbacks are critically endangered, yet the group from the Northwest Atlantic is currently considered to be under lower risk than other populations while hosting some of the largest rookeries. Here, we investigated the genetic diversity and the demographic history of contrasted rookeries from this group, namely two large nesting populations in French Guiana, and a smaller one in the French West Indies. We used 10 microsatellite loci, of which four are newly isolated, and mitochondrial DNA sequences of the control region and cytochrome b. Both mitochondrial and nuclear markers revealed that the Northwest Atlantic stock of leatherbacks derives from a single ancestral origin, but show current genetic structuration at the scale of nesting sites, with the maintenance of migrants amongst rookeries. Low nuclear genetic diversities are related to founder effects that followed consequent bottlenecks during the late Pleistocene/Holocene. Most probably in response to climatic oscillations, with a possible influence of early human hunting, female effective population sizes collapsed from 2 million to 200. Evidence of founder effects and high numbers of migrants make it possible to reconsider the population dynamics of the species, formerly considered as a metapopulation model: we propose a more relaxed island model, which we expect to be a key element in the currently observed recovering of populations. Although these Northwest Atlantic rookeries should be considered as a single evolutionary unit, we stress that local conservation efforts remain necessary since each nesting site hosts part of the genetic diversity and species history.

## Introduction

Natural populations are dynamic systems facing variations in time and space that are directly or indirectly related to environmental changes. Consequently, population genetics deals with non-equilibrium states, meaning that alongside long-term adaptive processes, other complex mechanisms have to be incorporated such as the balance of gene flows among populations, changes in the sizes of populations, population dispersals to gain new or depleted habitats, and movements between breeding and feeding areas. Among population dynamics models, the metapopulation concept has been extensively considered and refers to an assemblage of ephemeral interacting subpopulations (i.e. including emigration and immigration events) that persist over time in a dynamic balance of local declines and increases [1], [2]. The extent of these interactions defines the strict metapopulation model, consisting of successive stages of extinction and colonization of local subpopulations, irrespective of the demography of other populations [3]. In contrast, the island model considers a total population divided into subgroups, each breeding randomly within itself, but with some migrants removed from the entire group [4], [5]. In both cases, dispersions between populations result in gene flows that influence the genetic diversity of sources and sink populations [6], [7].

Metapopulation theory also addresses demography and structure of subpopulations, and thus their extinction probability [8]. Higher loss of heterozygosity with lower migration rates induces lower effective population size [9], [10]. Also, when a new population is established by a very small number of individuals from a larger population, founding events are source of genetic drift, with populations of different ages showing different levels of structuration according to colonization time [11].

Demographic events and migrations also result in contrasted signatures of genetic diversity. A decrease in the effective population size results in an excess of gene diversity at neutral loci, because the rare alleles that were lost contributed little to the heterozygosity of the ancestral population [12]. In contrast, recent population expansion and founder effect result in a heterozygosity deficit [13]. In respect to migratory behavior - a trait that integrates behavioral, physiological and morphological characters as well as life histories [14] - the spatial segregation of breeding and nesting sites may result in successive stages of mixing and isolation of genetic stocks. Migration makes the assessment of differentiation within sympatric and parapatric populations [15] and the investigations of demographic histories [13] more difficult to achieve.

A good understanding of the history, magnitude and drivers of past changes is necessary if we hope to adequately assess the current status of threatened species and populations and make future projections of their likelihood of extinction or recovery [16], [17]. The leatherback turtle (*Dermochelys coriacea,* Vandelli, 1761) is a pelagic marine species widely distributed in tropical and subtropical waters and is currently classified as ”critically endangered„ with a constantly declining global population trend [18]. Today, the Atlantic Ocean hosts most of the world's populations, some of them showing stable and even positive trends in terms of nesting activity [19]. Most of the largest Atlantic rookeries are located in the north-eastern part of South America/West Indies and in western Central Africa [20], considered as part of the Regional Management Unit (RMU) of the northwest Atlantic, and southeast Atlantic RMU, respectively [21]. The NW Atlantic RMU has been classified as ‘low risk’ and is considered to face low threats [22]. The leatherback turtle's life cycle involves pluriannual migrations after the nesting periods [23], [24] and female natal homing behavior [25], [26], and this complexity makes the issues of population dynamics and status difficult to address. Nevertheless, our understanding of phylogeographic patterns, population dynamics and behavior in sea turtles has been greatly improved thanks to molecular markers [26]–[32]. Autosomal microsatellite variability has been shown to provide relevant estimates of both the timescale and strength of past demographic events [33], [34] thus allowing the assessment of recent changes in population size and potential recovery [17], [35]. However, few studies using microsatellite markers have been performed on leatherbacks [28], [29]. No founder effect and/or bottlenecks were evidenced, and consequently a metapopulation model was suggested, with a rapid turnover of rookeries and settlements of new populations resulting from massive arrivals of a large number of migrants [29], [36].

In this study, we aimed to investigate the recent demographic history and the current fine-scale structure of the NW Atlantic Ocean RMU using the most recent markers, including some recently published [37], [38] and sensitive analytical methods [33], [39], [40]. We focused on three nesting rookeries that are very different in terms of population sizes and recent trends in nesting activities. Two of these rookeries are in French Guiana, namely (i) the historical major nesting site of Awala-Yalimapo, where thousands of nests have been recorded yearly for decades [20], [41], and (ii) the recent nesting site of Cayenne [42] where nesting activity increased from 3,000 nests to 9,000 nests/year during the last decade. The study is completed by the small nesting sites of Guadeloupe and Martinique (French West Indies) where only a few dozen females are observed every year [43]. We tested individuals within these rookeries for a set of 10 microsatellite markers, and sequenced the control region and the mtDNA cytochrome b gene to consider:

(i) The small-scale structure of these rookeries and the strength of migrations among the rookeries in order to achieve a precise evaluation of nest-site fidelity and geographic level of gene flow within the NW Atlantic RMU,

(ii) The historical baselines of effective population sizes, in order to understand the possible extent of recent demographic changes and their significance for current and future population status.

## Materials and Methods

### Field Sampling and DNA Storing

Skin biopsies (with Biopsy Punch 4 mm, Kruuse©, conserved in 99% ethanol), or blood samples (with a heparinised syringe in the venous sinus in the hind flipper) were collected from nesting leatherbacks during oviposition between 1990 and 2010. Three sets of samples were considered, and corresponded to the three following rookeries: (i) Awala-Yalimapo (AY), Western French Guiana, at the border with Suriname (n = 52); (ii) Cayenne (CAY), East French Guiana, 300 km east of AY (n = 95); and (iii): Martinique (n = 56) and Guadeloupe (n = 12) in the French West Indies (FWI), 200 km apart and 2,000 km northwest of French Guiana (Figure 1). Total DNA was extracted following the phenol/chloroform procedure [44].

**Figure 1:** Sampling sites and haplotype distribution of the control region (mitochondrial DNA) in the leatherback turtle, *Dermochelys coriacea.*

### Microsatellite standardization

We built two microsatellite enriched genomic libraries [45]. One of the libraries was enriched for dinucleotide sequences using (CT)_8_ and (GT)_8_ biotinylated microsatellite probes and the other for tetranucleotide sequences using (GATA)_4_ and (GACA)_4_ biotinylated microsatellite probes. The selected fragments were amplified by PCR then cloned into the pGEM-T vector (Promega©). Plasmids were introduced into XL-1 blue cells and transformed cells were cultivated on agar plates (incubation temperature = 37°C) containing 100 µg/ml of X-galactosidase and ampiciline. About 500 clones containing inserts were sequenced with the ET Dye terminator Cycle Sequencing Kit (Amersham Biosciences) following the manufacturer's recommendations for sequencing in an automated MegaBACE 1000 DNA analysis system. Repeated microsatellite motifs were found using the Gramene Project SSR tool [46]. 39 sequenced clones presented microsatellite motifs from which 14 primer pairs were designed and synthesized. For those 14 microsatellites, PCR conditions were optimized after the successive amplifications of five samples, and thereafter 32 samples were amplified to check putative genotyping errors, polymorphism and the quality of the peaks discriminating alleles. This procedure allowed us to identify four of the most informative markers, namely Dc003, Dc005, Dc008 and Dc013) (Table 1).

**Table 1:** New microsatellite primers for the leatherback turtle, *Dermochelys coriacea*. Ta - Annealing temperature; Repeat motif; Range of Fragment size (in base-pairs).

Locus	Primer sequence (5'-3')	Ta (°C)	Repeat motif	Range of Fragment size (bp)	A (n = 215)	AR (n = 215)
Dc003	F- 5'-AAGCCCTCAGCATTTGAAGT-3'	60	(ATCT)_12_	170–218	12	8.78
	R- 5'-CAATTTATCACAAAGATATCACC-3'					
Dc005	F - 5'-GGCCTTTGATGCAAGTAGGA-3'	54	(GT)_19_ (TC)_7_	183–205	9	4.35
	R - 5'-CAGGACTCACATAAAGTG-3'					
Dc008	F - 5'-AATTGGATGACGAGCAGGAC-3'	66	(GT)_20_	184–220	13	10.64
	R - 5'-GTCTCTCGCTGCCCACTGCTC-3'					
Dc013	F- 5'-ACCGGTGGCACCTTAGAGAC-3'	66	(AC)_13_	153–167	6	4.44
	R- 5'-CCAACAGAAGTATCACATCATGTTCTC-3'					

A–Total number of alleles; AR–Allelic richness;

### Microsatellite genotyping

Besides the four new markers developed in this study (see above), we also analyzed P186, Dc99 [47], Nigra32 [48], LB141 [37], Derm 5 and Derm 34 [38]. Part of the genotyping (Dc003, Dc005, Dc013, P186, LB141, Derm5 and Derm34) was performed on a Beckman Coulter automated sequencer, using pre-labeled primers with labels D2, D3 or D4. Polymerase chain reaction (PCR) mixes were performed in a 9 µl total reaction volume including 1 µl of genomic DNA (∼10 ng), 0.5 U of Taq polymerase (BioLine©), 200 µM of deoxynucleoside triphosphates, 1X Tris–KCl buffer, 1.0–3.0 mM MgCl_2_ (BioLine©), and 0.5 µM (for P186 and Nigra 200) or 1.0 µM of each primer. Other loci (Dc008, Dc99 and Nigra32) were analyzed using MegaBACE 1000, in which primers were synthesized with a M13 tail and fluorescent complementary sequences were added in the PCR reactions [49]. PCR conditions were the same, but in this case we used 0.3 U of Taq Platinum (Invitrogen©) and added 1.0 µM of the complementary M13 reverse primer and 0.1 µM of the forward primer, both labeled with FAM or HEX fluorescences. The amplification program for Dc008 consisted of 3 min at 94°C, followed by 10 cycles of 45 s at 94°C, 45 s at 66°C, 90 s at 72°C and 25 cycles of 45 s at 94°C, 45 s at 50°C, 90 s at 72°C, and a final extension step of 40 min at 72°C. For LB141, Derm5 and Derm34 we followed the conditions previously used by the authors. For the other markers, the amplification program consisted of 3 min at 94°C, followed by 30 cycles of 30 s at 94°C, 30 s at specific annealing temperature, 30 s at 72°C, and a final extension step of 30 min at 72°C.

### Mitochondrial DNA Markers

The mtDNA control region (CR) was entirely amplified for 68 samples (AY: n = 17, CAY: n = 22; FWI n = 29) using the primers LCM 15382 and H950 [50]. The cytochrome b (Cyt-b) gene was amplified for 102 samples (AY: n = 33, CY: n = 40, FWI: n = 29) using primers L595/Htr8 and L31Glu/H701 [51]. PCR mixes of 50 µL included 2 µl of genomic DNA (∼20 ng), 2 U of Taq polymerase (BioLine©), 200 µM of desoxynucleoside triphosphates, 1X Tris–KCl buffer, 3.0 mM MgCl_2_ (BioLine©), and 0.4 µM of each primer. The amplification program for both markers consisted of 10 min at 94°C, followed by 35 cycles of 30 s at 94°C, 30 s at 51°C for CR and at 55°C for Cyt-b, 1 min at 72°C, and a final extension step of 15 min at 72°C. PCR products were sent for sequencing to Beckman Coulter Genomics (Takeley, UK). The consensus and the sequences were aligned with Clustal W implemented in MEGA 5.05 [52], with manual edition when necessary. All sequences were deposited in the GenBank database (control region: JX629672 to JX629739; cytochrome b: KC354403–KC354442).

### Microsatellite data analysis

GIMLET software [53] was used to quantify genotyping errors for the 10 microsatellites by repeat-genotyping. We randomly selected approximately 25% of all samples (n = 47 individuals) and independently repeat-genotyped these four times for all loci. Across the four genotypings, averaged across loci and across samples, we detected low error values: 1.2% of dropout, 1,1% of false allele, 0.4%, 0.4%, 0.5%, 0.4% and 0.2% of type 1, type 2, type 3, type 4, and type 5 errors, respectively.

We checked for occurrence of linkage disequilibrium among the 10 microsatellite loci with GENEPOP 1.2 [54] and verified any presence of null alleles with MICROCHECKER 2.2.3 [55] and INEst 1.0 [56], the latter also making it possible to adjust genotype frequencies using the PIM estimator [57]. The Markov chain method was used to assess Hardy–Weinberg equilibrium and observed heterozygote excess of microsatellites, using GENEPOP 1.2. Nucleotide diversity was calculated with FSTAT 2.9.3.2 [58]. ARLEQUIN 3.5 [59] was used to calculate nucleotide diversity, to evaluate the differentiation among populations (RST and FST) and perform neutrality tests (Ewens-Watterson neutrality test and Chakraborty's amalgamation test). An asymmetric estimate of the migration rate between a subset of pairwise populations was calculated using MIGRATE 3.2.19 [60], with Bayesian inference strategy and single-step model. Initial runs were set estimating theta (Θ = 4Ne× µ, with Ne = effective population size and µ = mutation rate) and Nm (number of migrants) with FST, allowing Nm to be asymmetric. Reruns were set using the parameter estimate found in the first run and lengthening the Markov Chain Monte Carlo. MIGRATE 3.2.19 allowed to define not only emigration and immigration rates, but also their evolution and the evolution of theta and Nm through time.

A Bayesian clustering approach implemented in STRUCTURE 2.3.1 [61] was used to determine whether any hidden population structure resulting from distinct ancestral stocks could falsely generate a signature of population collapse [62]. This method uses a Markov Chain Monte Carlo (MCMC) approach in order to group individuals into K populations based on their genotypes without any prior information. We tested K  = 1to K = 10, using the admixture population model, 1,000,000 iterations, 50,000 burn-in replicates and five independent replicates per K value. The best K value was defined using the log probability of the data Pr(X | K) for each value of K [63].

We also used a multivariate method to make assumptions regarding data structure. Unlike STRUCTURE, multivariate models do not assume that populations are in Hardy-Weinberg equilibrium. Accordingly, a Discriminant Analysis of Principal Components (DAPC, [39]) was performed with the package *adegenet* in R 2.13.0 [64] in order to identify and describe sequence clusters. The DAPC relies on data transformation using Principal Component Analysis (PCA) as a prior step to Discriminant Analysis (DA), which maximizes the separation between groups. The optimal number of clusters was predicted using the sequential K-means clustering method, and the Bayesian Information Criterion (BIC) was used to choose the best number of groups (K) from 1 to 10.The number of clusters was assessed using the function *find.clusters*. In all analyses, 40 principal components (PCs) were retained, corresponding to the number of principal components that explained 90% of the cumulative variance.

We used MSVAR1.3 [40] to analyze the demographic histories of each leatherback rookery, the effective ancestral and current population sizes and time since collapse or expansion for each of them. A priori mutation rates of nuclear DNA ranging from 6×10^−4^ to 9.5×10^−3^ were previously set in several marine turtle species [65] for pre-runs, and posterior values of mutation rates after convergence were used for final runs. An exponential model was used [34]. The convergence was checked in TRACER [66] to ensure that all parameters had an Effective Sample Size (ESS) of at least 100. Generation time for leatherback ranges from 10 to 30 years [67]–[69]: demographic features were explored using an intermediate value of 16.1 years [69].

We also used the Extended Bayesian Skyline Plots (EBSP) [33] to estimate the population size through time. This method allows inference of the population demographic history by averaging over a nested set of microsatellite mutation models that incorporate length dependency, mutation bias and step size. We ran the analysis in BEAST v. 1.7.1 for 500,000,000 iterations, and parameters were sampled after every 5,000 iterations. The convergence was checked in TRACER [66] with ESS>100. Mutation rate and generation time were identical to those used for MSVAR estimates. The range of the mutation rate was set as a uniform distribution, and the mutation model was set as the Two-Step. We also modified the operators according to the EBSP tutorial (http:// http://beast.bio.ed.ac.uk). A preliminary analysis was performed using the Coalescent prior, and constant population size was also run in BEAST in order to estimate the population size. We used these results to set the population size prior in the EBSP analysis, using a uniform prior and the 95% CI estimated with the constant population size. In order to compare models and check if the EBSP results were different from a constant size model we calculated a Bayes Factor (i.e., the harmonic mean of the log likelihood [70]), and thus obtain support for one model over another, using both the EBSP and the constant population size prior.

### Mitochondrial DNA data analysis

Both CR and Cyt-b gene sequences were analyzed for haplotype and nucleotide diversities with DNAsp 4.20.2 [71]. Tests for differentiation between populations (FST, and Exact Test of Differentiation) as well as neutrality tests (Tajima's selective neutrality test, Ewens-Watterson neutrality test, Chakraborty's amalgamation test and Fu's neutrality test [72]) were performed with ARLEQUIN [59]. We used BEAST 1.7.1 to generate Bayesian Skyline Plots (BSP) [73] for an assessment of historical changes in the effective population size (*Ne*) over time. We applied a strict molecular clock and a piecewise-constant Bayesian skyline tree prior. A mutation rate of 2% per site per Million Years Ago (MYA) was considered [36].The most likely mutation model was estimated with MRMODELTEST [74]. Convergence was checked based on likelihood, as previously described.

## Results

### Microsatellite data

Since leatherbacks from AY had been sampled over a long period, two preliminary approaches were implemented in order to control a putative bias resulting from genetic drift during this period: (i) differentiation among rookeries was calculated using RST and FST indexes between 2 periods: samples collected in 1990–2000 vs. those collected in 2001–2010, and no structuration was evidenced; (ii) STRUCTURE was used to investigate the number of ancestral stocks within this sample. It revealed that a single stock (K = 1) was the most probable solution. Consequently, all the samples from AY were considered as a single rookery.

All the 10 microsatellite loci were polymorphic and linkage disequilibria were not significant (*p*>0.05) after Bonferroni correction. Regarding the 4 new microsatellite markers developed specifically for this study (Dc003, Dc005, Dc008 and Dc013), Dc008 presented the highest allelic richness (AR = 10.64, averaged among sample sets), while Dc005 presented the lowest allelic richness (AR = 4.35). The number of alleles per locus ranged from 4 (Nigra32) to 29 (LB141) (Table 1). Gene diversity (Gd) of Dc008 ranged from 0.82 in AY to 0.84 in CAY rookery, with similar diversities among sampling rookeries (Table 1). Considering all loci, gene diversities were comparable in CAY and FWI rookeries, and slightly lower in AY (Table 2). Dc008 presented null alleles in CAY and FWI rookeries, Derm34 and LB141 presented null alleles in AY rookery.

**Table 2:** Microsatellite diversity indexes for the leatherback turtle, *Dermochelys coriacea*, for each rookery and each marker: Gd - Gene diversity, He - Expected heterozygosity, Ho - observed heterozygosity (Ho), FIS - inbreeding coefficient (FIS).

Locus	Gd			He			Ho			FIS		
	CAY	FWI	AY	CAY	FWI	AY	CAY	FWI	AY	CAY	FWI	AY
Dc003	0.78	0.76	0.78	0.77	0.76	0.79	0.74	0.83	0.86	0.039	−0.109	−0.100
Dc005	0.45	0.56	0.49	0.45	0.55	0.49	0.43	0.51	0.45	0.044	0.086	0.088
Dc008	0.84	0.84	0.82	0.84	0.84	0.82	0.69	0.72	0.75	0.176	0.145	0.076
Dc013	0.39	0.41	0.14	0.39	0.41	0.14	0.37	0.40	0.15	0.044	0.016	−0.053
LB141	0.77	0.84	0.81	0.77	0.81	0.83	0.72	0.75	0.65	0.061	0.073	0.220
Derm5	0.79	0.78	0.82	0.79	0.79	0.82	0.75	0.74	0.81	0.057	0.066	0.012
Derm34	0.93	0.92	0.88	0.93	0.92	0.87	0.89	0.90	0.82	0.042	0.024	0.295
Nigra3	0.64	0.66	0.69	0.64	0.66	0.69	0.60	0.69	0.69	0.060	−0.046	−0.007
Dc99	0.71	0.68	0.70	0.70	0.68	0.82	0.65	0.71	0.76	0.075	−0041	0.114
P186	0.60	0.60	0.61	0.60	0.60	0.61	0.58	0.56	0.61	0.036	0.064	−0.012

CAY: Cayenne, AY: Awala-Yalimapo, FWI: French West Indies.

The analysis of stocks using STRUCTURE indicated that the most probable number of populations (K value) was 1, therefore failing to recover any ancestral structure. The DAPC results were similar, and although the lowest value of BIC indicated a K = 6 (with a possible range from K = 3 to 7), individuals from all three sample sites were assigned in all six groups. Therefore DAPC also suggested a single ancestral stock.

When analyzing all ten loci with model genotypes that were either original or adjusted with PIM model [64], RST was only significant between CAY and AY (RST = 0.0289, p<0.05). However when excluding the three loci with null alleles, RST was significant between AY and FWI (RST = 0.0106, p<0.05), and between CAY and FWI (RST = 0.0211, p<0.05). FST provided a stronger structuration signal and was significant between the 3 rookeries with the 10 loci dataset, but not significant between CAY and AY only with the 7 loci (Table 3). According to AMOVA more than 98% of the genetic variation was within populations, while less than 2% was between populations.

**Table 3:** Structuration coefficients for the leatherback turtle, *Dermochelys coriacea*: RST (first values) and FST (second values) for each population pair, assessed from microsatellite markers in leatherback turtles sampled in rookeries in French Guiana (Awala-Yalimapo: AY, and Cayenne: CAY) and French West Indies (FWI).

	CAY	AY	FWI
CAY		0.02891*/0.007*	0.00908/0.018*
AY	−0.1965/0.003		0.01451/0.023*
FWI	0.02110*/0.02*	0.01064*/0.02*	

Above diagonal: analysis with 10 loci; below diagonal: analysis with the seven loci that did not present null alleles.

* Significant values (p<0.05)

Observed and expected heterozygosities, and Inbreeding coefficients, are shown in Table 2 for each locus and each population. None of the populations in original and adjusted genotypes in any of the ten microsatellite loci were in Hardy-Weinberg equilibrium, and all of them presented heterozygote deficit (Table 4). However, all of the populations were in Hardy-Weinberg equilibrium, when the loci with null alleles were excluded. According to analysis of ten microsatellites, AY has the highest inbreeding coefficient (FIS = 0.080) and gene diversity over loci (Gd = 0.732 respectively), while FWI has the lowest FIS (0.029) and CAY, and the lowest Gd over loci (0.677) (Table 4). When the three loci with null alleles are excluded, CAY presented the highest FIS (0.052) and FWI the lowest (0.001).

**Table 4:** Nuclear DNA diversity indexes for the leatherback turtle, *Dermochelys coriacea*, expected heterozygosity (He), observed heterozygosity (Ho), inbreeding coefficient (FIS), and MSVAR1.3 estimations of ancestral and current population sizes, and time since declines for leatherback turtle rookeries sampled in French Guiana (Awala-Yalimapo - AY and Cayenne - CAY) and French West Indies (FWI).

	He	Ho	FIS	Average gene diversity over loci*	Estimated Ancestral population size*	Estimated current population size*	Time since decline (years)*
CAY	0.689	0.644	0.066	0.677+/−0.355	2,500,000 [2,400,000–3,000,000]	250 [230–300]	11,000 [8,200–13,500]
AY	0.676	0.622	0.080	0.732+/−0.396	3,500,000 [3,300,000–4,900,000]	70 [66]–[78]	3,200 [3,100–3,900]
FWI	0.701	0.680	0.029	0.687+/−0.360	130,000 [120,000–144,000]	81 [75]–[89]]	2,880 [2800–3,650]

* mean [mean−SD/mean+SD]

We found a high rate of gene flow among rookeries, with 13 to 33 migrants per generation (between FWI and AY, and between CAY and AY, respectively). In analyses which excluded the loci with null alleles, the number of migrants between AY and CAY was seen to increase to 80, whereas it remained in the same range (12) between AY and FWI. Whatever the set of data used, emigrants from CAY and FWI to AY were twice as numerous as immigrants from AY to other rookeries.

Sensitive Bayesian methods implemented in MSVAR showed dramatic declines in effective population sizes, with ancestral effective population sizes ranging from 120,000 (Awala-Yalimapo) to 1,600,000 (CAY) shrinking to current effective population sizes ranging from 70 (FWI) to 120 (CAY) (Figure 2). This corresponds to a decline of 99.99%, leaving a total effective population size around 500–1,500 females for each rookery (Figure 3). These bottlenecks occurred at two periods, namely around 2,000 to 3,500 YA for AW and FYI, and earlier (10,000 YA) for CAY (Figure 3). MIGRATE revealed a slight increase of theta in all three rookeries 100–200 YA, suggesting low but increasing effective population sizes, which is congruent with MSVAR results (Figure 3). Unlike the above mentioned tests, the Extended Bayesian Skyline Plot (EBSP) graph shows a flat line for all the three rookeries through time, with a fast recent increase less than 20 generations ago (Figure 3). Yet, when the Bayes Factor (BF) was calculated for the EBSP and assuming a constant population size model for each rookery, the simplest coalescent model performed better in comparison to the EBSP (log_10_ BF>30). The sizes of populations estimated with the constant coalescent model were concordant with MSVAR analysis, indicating three small effective populations of approximately 100 females. Additionally, by the parameter onePhaseProb revealed that a low occurrence of microsatellites mutating as a single step (ranging from 0.14 to 0.16), indicating that in the most cases the loci analyzed do not follow the single step mutation model, but rather change length in a>1 repeat unit.

**Figure 2:** Posterior distributions of highest posterior density intervals for current (N0) and historic (N1) estimates of effective population size with three independent runs of MSVAR1.3, for the leatherback turtle, *Dermochelys coriacea* from three rookeries: Cayenne (CAY), Awala (AY) and French West Indies (FWI).

**Figure 3:** Recent demographic histories of the northwest Atlantic leatherback turtle *Dermochelys coriacea* from three rookeries of Cayenne, Awala-Yalimapo (French Guiana) and Martinique/Guadeloupe (French West Indies), based on microsatellite analysis, using (i) MSVAR (up), (ii) MIGRATE, (middle), and (iii) EBSP (down).

### Mitochondrial DNA data

Regarding the CR (711 bp), a total of five haplotypes were evidenced, all of which were present in AY, with Dc_A5 and Dc_C3 being newly reported and exclusive of this rookery. All three rookeries shared the other three haplotypes, revealing the presence of Dc_C2 for the first time (Figure 1, Table 5). The structuration coefficient of (FST) was low but significant between CAY and FWI (FST = 0.0955, p = 0.045) and between AY and FWI (FST = 0.0995, p = 0.037) (Table 6). An exact test of differentiation showed significant differences between AY and CAY (p<0.05), and AY and FWI (p<0.05), but not between CAY and FWI (p>0.05). AY presented the largest gene diversity (Gd = 0.794), showing all five CR haplotypes. FWI was the rookery displaying the lowest gene diversity (Gd = 0.352) (Table 7). None of the rookeries showed any deviation of neutrality according to Tajima's selective neutrality, Ewens-Watterson neutrality, Chakraborty's amalgamation and Fu's neutrality tests. Full Cyt-b sequences (1,111 bp) showed very low variability, with only two haplotypes differentiated by one polymorphic site, both present in the three rookeries. There is no evidence of population structure and, in this case, gene diversities were low (Gd ranging from 0.340 to 0.492). The Bayesian Skyline Plot was inferred with the CR only, since the Cyt-b showed extremely low levels of variability. The most probable substitution model was HKY with invariant sites; BSP failed to show any significant change in population size over the last 12 MYA, but this result should be interpreted with caution given the low variability observed in this gene.

**Table 5:** mtDNA control region polymorphisms and haplotype designations for the leatherback turtle, *Dermochelys coriacea* rookeries sampled in French Guiana and French West Indies (FWI) associated to 496 bp [36] and 711 bp [32].

	Base position											
496 bp haplotypes	150	215	228	246	259	308	622	632	690	694	703	711 bp haplotypes
Dc_A	G	A	G	T	G	A	A	A	C	T	T	Dc_A1
Dc_A5	.	.	.	G	.	.	.	.	.	.	.	Dc_A5
Dc_C	A	G	A	.	.	G	.	G	.	.	.	Dc_C
Dc_C	A	G	A	.	.	G	.	G	.	C	.	Dc_C2
Dc_C3	A	G	A	G	.	G	.	G	.	C	.	Dc_C3

Polymorphisms from positions 150 to 308 are also included in the 496 bp haplotypes.

**Table 6:** Pairwise FST based on control region (Mitochondrial DNA) for for the leatherback turtle, *Dermochelys coriacea* rookeries sampled in French Guiana (Awala-Yalimapo - AY and Cayenne - CAY) and French West Indies (FWI).

	CAY	AY	FWI
CAY	0.000	0.036	0.096*
AY		0.000	0.099*
FWI			0.000

* significant values (p<0.05)

**Table 7:** Diversity of mtDNA control region for for the leatherback turtle, *Dermochelys coriacea* rookeries sampled in French Guiana (Awala-Yalimapo - AY and Cayenne CAY) and French West Indies (FWI).

	Sample size	No of haplotypes	Gene diversity (mean+/−SD)	Nucleotide diversity (mean+/−SD)
CAY	22	3	0.623+/−0.073	0.0041+/−0.0025
AY	17	5	0.794+/−0.061	0.0047+/−0.0028
FWI	29	3	0.352+/−0.098	0.0025+/−0.0017

## Discussion

Leatherback turtles exhibit complex life traits, including female homing and migration, migration patterns of juveniles that remain little known to date, and climate that has been shown to strongly influence resources, breeding success and sex-ratio. Based on a comprehensive integrated approach combining microsatellite and mitochondrial DNA, our study provides new insights into the population dynamics of leatherbacks in the Northwest Atlantic, considered as one of the world's largest populations [20], with significant recovery potential [75]. Our genetic data are expected to contribute to a better understanding of their history and current dynamics, and ultimately play a part in their conservation.

### Methodological issues

This work puts forward the complexity of analytic choices with concurrent approaches. We used three methods based on Bayesian inference, namely MSVAR, BEAST and MIGRATE, to explore recent demographic history and changes in the evolution of effective population size in distant rookeries with contrasted numbers of nesting females. MSVAR has been shown to be a relevant tool to detect expansions and declines in different species [34], including sea turtles [17]. Bottlenecks of variable extent and dates were detected by MSVAR, but not by the EBSP method. However, to our knowledge this is the first time the EBSP method has been used with data from natural populations, and thus precludes further analysis of the comparative sensitivity of these methods. Interestingly, all three approaches identified low and congruent values of current effective population sizes, and the very recent expansion signal detected by MIGRATE is indicative of populations recovering after bottlenecks.

One other key point in our study was a high estimated occurrence of null alleles in our dataset. Null alleles result in lower heterozygosity and consequently impact the structuration signal among populations, overestimating the distances among clades [76]. The recent adaptation of the PIM model [57] makes it possible to assess inbreeding coefficients and allele frequencies with a high level of confidence [64]. In our study however, the use of our full dataset, including loci without null alleles and loci with corrected frequencies, resulted in lower structuration among rookeries than when only loci without null alleles were used. Consequently, as observed in other endangered species [77] and confirmed by the low rate of genotyping errors, we conclude that a true homozygote excess has resulted from low population sizes, inbreeding and genetic drift [78], rather than a high occurrence of null alleles.

### Fine scale population structure and genetic diversities

The concurrent use of different methods to analyze sequences of the control region and autosomal microsatellite variability in this study has revealed that the Northwest Atlantic stock of leatherback turtles derives from a single ancestral origin, but shows a current genetic structure at a small geographic scale that is related to the distribution of nesting rookeries.

The sequencing of the entire Cyt-b revealed evidence of only two haplotypes, probably the same as those previously described and based on shorter sequences (876 bp) [79]. But despite those longer sequences, a signal of limited structure was evidenced, reinforcing the idea of a wide North Atlantic stock [36]. Analysis of the control region, a more variable gene, revealed the signature of some structure between French Guiana and French West Indies, which contrasts with the previous study showing the presence of only one 496 bp haplotype in the Guianas and three haplotypes in the West Indies [36]. These differences could be explained by the longer sequences used in this study, hence improving the resolution of mtDNA for comprehensive phylogeographic studies [32].

Among our five CR haplotypes, only two have been previously described [32], [36]. Our large sample set also enabled a significant increase in the diversity indexes of the Northwest Atlantic Leatherback populations, contrasting with the first assessments made [36], and resulting in the highest diversities reported in the species along with Indo-Pacific nesting populations [32]. The highly sensitive microsatellite markers revealed low, small-scale structuration that was also observed between the Awala-Yalimapo and Cayenne rookeries despite the short distance between these two sites (<300 km).This pattern could seem intriguing, considering the very long distance and the behavioral plasticity of the leatherback during its pluriannual migrations [20], [23], [75], [80], [81], but supports the argument for fidelity to nesting sites [25], [26].

### Late Pleistocene and Holocene demographic changes

Microsatellite markers revealed a low genetic diversity compared to other marine turtle species [82], [83]; this is probably related to their recent demographic histories. Our results indicate that the North Atlantic population of leatherbacks experienced bottlenecks in the Late-Pleistocene and Holocene, with two major events, in 12,000 YA and from 3,500 to 2,000 YA. Ancestral size of effective population collapsed from 120,000–1,500,000 females, falling to the present estimations of 70 (AY) to 250 (CAY) females for each rookery. The population declines we found for the north Atlantic leatherback were of similar magnitude than those reported in the north Atlantic olive ridley turtle (*Lepidochelys olivacea*) [17], the green *Chelonia mydas* and the hawksbill *Eretmochelys imbricata* turtles in the wider Caribbean region [84], as well as marine mammals [35], [85], [86]. Most of these declines are assumed to have occurred in the Holocene and have to be considered as a widespread pattern in the large vertebrate populations of the North Atlantic.

Following the idea of recent megaufauna extinction and the controversial ”blitzkrieg„ hypothesis [87] collapses in leatherback populations could be attributed to human interactions such as historical egg poaching, selective harvesting and hunting [19], [35], [84]. The collapses may also be the result of previous climate oscillations during the Holocene [88]–[90]. Fine-scale differences in the use of feeding areas, and/or distinct behavioral patterns [75] may explain why the rookeries were not affected concomitantly. Environmental conditions may impact marine turtles either directly by harming females and hatchlings, and affecting temperature-dependent sex-ratio [91], or indirectly by affecting nesting beach quality and availability [92], the ability of oceanic-driven hatchlings to home to their birth site [93], and trophic conditions in foraging areas [94], [95].

### Population dynamics models

The recovery of populations suggested by both recent increases of effective population sizes and positive trends of nesting activities [20] will be influenced by population dynamics models [8]. Although the population dynamics of leatherbacks has been extensively discussed on the basis of capture/mark/recapture data [review in 20], little attention has been paid to this question in relation to high resolution genetic data [36]. A metapopulation model has been accepted for the Atlantic [29] and western Pacific populations [96], considering that settlements of new populations would result from massive arrivals of a large number of migrants. Previous results support this idea, illustrating the absence of signatures for founder effects and/or bottlenecks [29]. A different approach to these results is now possible thanks to the use of new markers and more powerful methods of analysis to identify these signatures.

Metapopulation functioning implies that some groups are separated by habitat types that are not relevant for feeding and/or breeding activities [2]. In the case of the leatherback, it seems that such patterns are driven by nesting activity, due to the phylopatry of nesting females [25] rather than by feeding areas. However, structuration index values remain low despite significant small-scale structure, and high numbers of migrants are observed. Thus, leatherbacks may be driven by an island model rather than a strict metapopulation model that would imply successive cycles of extinction and recolonization [4]: in response to ecological opportunities, demes size would locally increase and decrease, but maintaining gene flow among demes. Emigrant and immigrant rates provide further information on the dynamics of the Northwest Atlantic Leatherback Turtle population. The CAY rookery, despite lower diversity, displays a higher number of emigrants than immigrants arriving from the two other rookeries. Higher population sizes, resulting from the recent expansions, may favor dispersal of breeders. All the methods used showed that current effective population sizes in the three rookeries were rather low, and no relationship with nuclear and mitochondrial genetic diversities was found. It can be suggested that the high number of migrants is associated with males rather than females, but this cannot be certified without further studies of male-mediated gene flow and its contribution to population dynamics and diversity.

Although the metapopulation theory implicitly refers to non-migrating species, this model has also been explored in migrating species, and namely in birds [8]. The leatherback thus represents an exciting new model to investigate the impact such behavioral traits could have on the genetic structure of populations.

### Conservation issues

Assessments of genetic diversity based largely on neutral variation provide essential information about population history and demography [97]. The Regional Management Units of the leatherback, up to and including the suggested geographic limits of the populations, are mainly managed using nesting population evaluations, information gained from pit-tags, satellite tracking and previous genetic assessment of structure using markers with low resolution [21]. Here we highlight fine-scale structure, and the importance of every single nesting rookery that hosts its own richness despite the dispersal of animals during their transoceanic migrations [98]. Efficient conservation programs should then focus not only on shared areas used during long-distance migration [81], [99], but also on each nesting rookery harboring a specific nuclear genetic signature.

Maintaining a high level of genetic diversity is assumed to be essential for the conservation of viable populations [100]. However, some species with historical low genetic diversity, no doubt due to cycles of bottlenecks and expansions, are not necessarily endangered [101]. Thus, as soon as an island model is assumed, the maintenance of high number of migrants among rookeries could ensure the future of populations [102], [103], despite the low nuclear diversity and low effective population sizes. In the French West Indies and French Guiana, nesting activity showed clear positive trends, as also reported in the Wider Carribbean [104]. To some extent, this trend can be explained by ongoing conservation efforts [105], the biological and ecological characteristics of the species [75] and island population dynamics that enhance the ability of the leatherback species to recover from population oscillations related to changing environmental conditions.
